The article "Ginsenoside Rg1 Suppresses Non-Small-Cell Lung Cancer via MicroRNA-126-PI3K-AKT-mTOR Pathway" was retracted in 2023. Reasons: signs of a paper mill; compromised peer review; unreliable results or conclusions.

# Ginsenoside Rg1 Suppresses Non-Small-Cell Lung Cancer via MicroRNA-126-PI3K-AKT-mTOR Pathway

**DOI:** 10.1155/2022/1244836

**Published:** 2022-07-01

**Authors:** Panfeng Chen, Xiaoping Li, Xi Yu, Min Yang

**Affiliations:** ^1^Department of Respiratory and Critical Care Medicine, Tianjin First Central Hospital, Tianjin 300192, China; ^2^Department of Thoracic Surgery, Tianjin First Central Hospital, Tianjin 300192, China

## Abstract

As one of the most common cause of cancer death in the world, lung cancer causes approximately 1.6 million deaths annually. Among them, NSCLC accounts for approximately 85% of patients in whole lung cancer patients. Ginsenoside Rg1 has been confirmed to play an important role in various diseases including cancer. As one of miRNAs, miR-126 closely involves in pathogenesis of the several types of cancers including colorectal, prostate, bladder and gastric cancer, and so on. Thus, the present study aims to investigate effects of the Ginsenoside Rg1 on NSCLC and underlying mechanism. In the study, two lung cancer cell lines including A549 and H1650 were used. It was found that expression of miR-126 was decreased in PBMC of NSCLC patients compared to healthy control. Expression of miR-126 was decreased in cancer tissue compared to paracancerous tissues in NSCLC patients. Importantly, it was found Ginsenoside Rg1 could inhibit growth of lung cancer cells. miR-126 KD remarkably increased the expression of apoptosis genes including caspase 3 and caspase 9 and decreased cell viability in lung cancer cells including A549 and H1650 cells. Interesting, *in silico* analysis indicated that miR-126 could target PI3K signaling pathway, which was confirmed by WB assay. KD of PI3KR2 compromised promotion of miR-126 on cell apoptosis. Similarly, it was found that KD of mTOR compromised promotion of miR-126 on cell apoptosis. Inhibition of Ginsenoside Rg1 on growth of lung cancer cells was through miR-126 and mTOR. Thus, the present study confirmed that Ginsenoside Rg1 remarkably inhibit lung cancer, which is through microRNA-126-PI3K-AKT-mTOR pathway.

## 1. Introduction

Lung cancer is the most common cause of cancer death all over the world, which annually causes approximately 1.6 million deaths [1]. There are two distinct categories of lung cancer including non-small-cell lung cancer (NSCLC) and small-cell lung cancer (SCLC) according to histological classification [2]. Among them, NSCLC accounts for approximately 85% of patients in whole lung cancer patients [2]. The pathogenesis of lung cancer is multiple, mainly including tobacco smoking (accounting for more than 80% of cases), environmental pollution, genetics, and so on [3]. Lung cancer is also a molecularly heterogeneous disease, which makes it difficult to fully understand its biology [3]. The empirical use of cytotoxic therapy based on a physician's preference is the traditional therapy to treat lung cancer, which has moved to personalized medicine according to the genetic alterations of the tumour and the status of programmed death ligand-1 (PD-L1), which predicts for benefit from targeted therapies or immune checkpoint blockers (ICBs) [4]. A better understanding about the disease plays an important role in developing effective therapies to treat lung cancer.

The article "Ginsenoside Rg1 Suppresses Non-Small-Cell Lung Cancer via MicroRNA-126-PI3K-AKT-mTOR Pathway" was retracted in 2023. Reasons: signs of a paper mill; compromised peer review; unreliable results or conclusions.

In China, lung cancer is one of the most severe cancer types, causing a large number of deaths. In fact, the peak of morbidity and mortality caused by lung cancer has never fallen. The number of new cases of lung cancer is about 326,600 and the death number due to lung cancer is about 569,400 in a year in China [5]. Similar to other regions in the world, NSCLC accounts for 85% of all lung cancer cases [6].

*Panax ginseng* (C.A. Meyer) is one of the species that has been commonly used as a tonic in Eastern Asia for thousands of years [7]. Ginsenosides (GS), the bioactive compounds in Panax ginseng, have received more attention recently [8]. Ginsenosides have been demonstrated to exert an essential role in various diseases including inflammation [9] and cancer [10].

Micro-RNAs are a great family of small noncondign ribonucleic acid molecules (RNAs), among, as an important member of this family, microRNA-126 (miRNA-126 or miR-126) is encoded by 7^th^ intron of the EGFL7 gene in human chromosome 9q34.3 and expressed in many humans cells such as cardiomyocytes, endothelial, and lung cells [11]. miR-126 is reported to have several important physiological functions; for example, it is found to bind directly to the DNA, preventing the transcription, translation and degradation of mRNA [12]. miR-126 plays vital roles in several immune-related diseases [13]. MiR-126 is reported to mediate brain endothelial cell exosome treatment-induced neurorestorative effects after stroke in type 2 diabetes mellitus mice [12]. MiR-126 can facilitate vascular remodeling and decline fibrosis, and thus it is considered to be an important factor in the pathogenesis of cardiovascular diseases and cerebral stroke [11]. Importantly, miR-126 is closely involved in the pathogenesis of cancers. The expression of miR-126 is found to be reduced in colorectal, prostate, and bladder and gastric cancer [14]. A similar phenomenon was found in lung cancer cell lines [15]. Thus, miR-126 may be highly involved in the pathogenesis of lung cancer.

The PI3K (phosphatidylinositol-4,5-bisphosphate 3-kinase)-Akt (protein kinase B)-mTOR (mammalian target of rapamycin) signaling pathway is a signal transduction pathway involved in the regulation of multiple cellular functions including cell proliferation, survival, differentiation, adhesion, motility, and invasion, which is one of the most frequently dysregulated pathways in human cancers [16]. The PI3Ks are a family of related intracellular signal transducer enzymes capable of phosphorylating the 3 position hydroxyl group of the inositol ring of phosphatidylinositol (PtdIns) [17]. As a member of the phosphatidylinositol 3-kinase-related kinase family of protein kinases, mTOR plays an important role in cancer [18]. PI3K/mTOR pathways play an important role in the pathogenesis of NSCLC. In fact, inhibitors of PI3K signaling have been suggested as potential therapeutic agents in NSCLC [19]. Interestingly, it is found that miR-126 can improve the viability, colony formation, and migration of keratinocytes HaCaT cells by regulating the PI3 K/AKT signaling pathway [20].

The article "Ginsenoside Rg1 Suppresses Non-Small-Cell Lung Cancer via MicroRNA-126-PI3K-AKT-mTOR Pathway" was retracted in 2023. Reasons: signs of a paper mill; compromised peer review; unreliable results or conclusions.

In the present study, we investigated the expression of miR-126 in healthy and NSCLC patients and the effects of miR-126 on the growth of lung cancer cells. The effects of GS on lung cancer cells and the underlying mechanism were explored.

## 2. Materials and Methods

### 2.1. Serum and Tissue Samples

NSCLC patients (*n* = 81) and healthy controls (*n* = 81) were recruited from the Tianjin First Central Hospital. After obtaining written informed consent from these subjects, blood samples were collected to obtain serum samples by centrifugation. The serum samples in cryopreservation tubes were treated with liquid nitrogen and stored at − 80°C conditions. For lung tissue samples, 30 paracancerous and cancer samples were collected from NSCLC patients using the needle biopsy method. This study design obtained the approval of the Ethics Committee of Tianjin First Central Hospital (TJFCH 200101-TJ).

### 2.2. Cell Lines

Human NSCLC cells including A549 and H1650 were purchased from Procell Biotechnology (Wuhan, China). A549 and H1650 were cultured according to the manufacturer's instructions. Briefly, A549 and H1650 cells were cultured in RPMI1640 (Thermo Fisher, Catalog number: 61870036) supplemented with 10% exosomes-free FBS (Thermo Fisher, Catalog number: 10082147) at 37°C incubators containing 5% CO_2_. Cells were subcultured when confluence reaches more than 90%.

### 2.3. RNA Isolation and Quantitative Real-Time Polymerase Chain Reaction (qRT-PCR)

Total RNA was separated from A549 and H1650 cells using the Beyozol total RNA isolation reagent (Beyotime, Beijing, China).In brief, 500 *μ*L of each sample was incubated with 500 *μ*L Beyozol total RNA isolation reagent and incubated for 2 min at room temperature, followed by vigorous mixing. Then, samples were added to the RNA isolation column according to the protocol. Finally, RNA was dissolved in 20 *μ*L RNase-free water. The quality of the RNA was determined by NanoDrop 2000 (Thermo Fisher Scientific). Then, cDNA was transcribed from 500 ng of total RNA using BeyoRT™ II cDNA synthesis kit (Beyotime, Catalog number: D7170M, Beijing, China).

The article "Ginsenoside Rg1 Suppresses Non-Small-Cell Lung Cancer via MicroRNA-126-PI3K-AKT-mTOR Pathway" was retracted in 2023. Reasons: signs of a paper mill; compromised peer review; unreliable results or conclusions.

For qRT-PCR, it was performed on the Applied Biosystems real-time PCR ecosystem (Thermo Fisher, USA) using BeyoFast™ SYBR Green qPCR Mix (2x) (Beyotime, Catalog number: D7260-1 ml, Beijing, China). The assay was carried out in a total volume of 25 *μ*L reaction mixture containing 12.5 *μ*L BeyoFast™ SYBR Green qPCR Mix, 2 *μ*L of cDNA, 1 *μ*L of each primer, and 8.5 *μ*L RNase-free water. The optimized cycling conditions were as follows: initial denaturation at 95°C for 10 s, followed by 40 cycles of denaturation at 95°C for 10 s, and primer annealing and extension at 56°C for 30 s. Fluorescence signals were recorded at the end of each cycle. A melt curve analysis was measured following amplification to confirm the specificity of the amplified products. Melting curve analysis consisted of 65°C for 5 s, followed by an increase in temperature to 95°C for 5 s with continuous fluorescence reading. RNase-free water, 5x reaction buffer, dNTP, RNasin Ribonuclease inhibitor, and BeyoFast™ SYBR Green qPCR Mix. The relative expression was calculated using the 2^−ΔΔCt^ method with GAPDH as the internal reference. The primers sequences are exhibited in Table 1.

### 2.4. Western Blot

The protein levels of several genes were quantified by western blot. Briefly, total proteins were extracted using RIPA Lysis (Beyotime, Catalog number: P0013C, Beijing, China) according to the manufacturer's protocols. Then, proteins were isolated by 10% SDS-PAGE and electro-transferred on PVDF membranes (Bio-Rad, Hercules, CA, USA). Subsequently, the membranes containing proteins were seriatim incubated with the primary and secondary antibodies for the indicated time, including Phospho-PI3K p85/p55 (Tyr458, Tyr199) Monoclonal Antibody (PI3KY458-1A11, Thermo Fisher), PI3K p85 alpha Monoclonal Antibody (A3-D0) (Catalog #MA5-32917, Thermo Fisher), mTOR Antibody (#2972, Cell Signaling Technology), Phospho-mTOR (Ser2448) (D9C2) XP® Rabbit (mAb #5536, Cell Signaling Technology) and anti-GAPDH (ab8245; Abcam). The second antibodies are goat anti-mouse/rabbit (ab205719 and ab205718; Abcam). The protein signals were visualized using the ECL Western Blotting Substrate (Bio-Rad) and quantified using Image J software (NIH, Bethesda, MA, USA).

### 2.5. Immunohistochemical Staining (IHC)

Immunohistochemical staining was carried out with the standard immunohistochemistry protocol. In brief, processed sections were incubated with anti-Phospho-PI3 Kinase p85 (Tyr458)/p55 (Tyr199) (E3U1H) (Rabbit mAb #17366, Cell Signaling Technology). Brown cytoplasmic staining is represented as the positive expression of those factors.

The article "Ginsenoside Rg1 Suppresses Non-Small-Cell Lung Cancer via MicroRNA-126-PI3K-AKT-mTOR Pathway" was retracted in 2023. Reasons: signs of a paper mill; compromised peer review; unreliable results or conclusions.

### 2.6. MTT Assay

A549 and H1650 cells were plated into a 96-well plate at a density of 5 × 103 cells/well and cultured in an incubator at 37°C supplemented with 5% CO_2_. After culturing for 48 h, 10 *μ*L MTT solution (Catalog number: C0009S, Beyotime, Beijing, China) was added into each well, incubating for another 2 h. Then, DMSO was added to remove formazan. The value of optical density (OD) in each well at 570 nm was measured using a microplate reader (Thermo Fisher Scientific; Waltham, MA, USA).

### 2.7. siRNA Transfection

24-well plates were used for seeding cells that were subjected to transfection with either siRNA (0.4 *μ*g) vectors including miR-126 mimics, miR-126-siRNA, PIK3R2-siRNA (silencing vector for PIK3R2, p-GPU6-PIK3R2-shRNA), mTOR-siRNA, and siRNA control (scramble). Transfections were performed according to the instructions for Lipofectamine 2000 (Invitrogen, USA), and 48 hours later, further analysis was performed.

### 2.8. Statistical Analysis

The data were analyzed using GraphPad Prism software (v8.0; GraphPad Prism, La Jolla, CA, USA) and shown as mean ± Standard error of the mean. Data comparison was conducted by using Student's *t*-test or analyses of variance (ANOVA) with Tukey post hoc test. *P* value less than 0.05 was regarded as statistically significant.

## 3. Results

### 3.1. The Expression of miR-126 Was Downregulated in PBMC and Lung Tissue of NSCLC Patients

To investigate whether miR-126 is involved in the pathogenesis of NSCLC, expression of miR-126 in PBMC of NSCLC patients (*n* = 81) and healthy controls (*n* = 81) was measured. It was indicated that the expression of miR-126 was significantly lower in NSCLC compared to healthy control (*P* < 0.001, Figure 1(a)). The expression of miR-126 in lung cancer needle biopsies and paracancerous tissues was investigated, which indicated that expression of miR-126 was significantly higher in lung cancer tissues than in lung paracancerous tissues (*P* < 0.001, Figure 1(b)). Thus, it was confirmed that expression of miR-126 was higher in the PBMC of NSCLC patients than in healthy controls, and it was higher in lung cancer tissue than in paracancerous tissues in NSCLC patients.

### 3.2. Knockdown (KD) of miR-126 Induced Apoptosis of A549 and H1650 Cells

Biogenesis of NSCLC, the expression of miR-126 in lung cancer needle biopsies and paracancerous tissues, two miR-126 vectors miR-126 vectors (#1 and #2), and a control vector (siRNA-scramble) were transfected in A549 cells, which indicated that both miR-126 vectors significantly increased the expression of the caspase 3 in A549 cells (^*∗∗*^*P* < 0.01, *n* = 4, Figure 2(a)). Moreover, it was found that both miR-126 vectors significantly increased expression of caspase 9 in A549 cells (^*∗∗*^*P* < 0.01, *n* = 4, Figure 2(b)). In addition, it was found that two miR-126 vectors significantly decreased the growth of A549 cells (^*∗∗∗*^*P* < 0.001, *n* = 6, Figure 2(c)). To further validate the effects of miR-126 on the growth of lung cancer cells, another NSCLC cell line named H1650 was used. Two miR-126 vectors (#1 and #2) and a control vector were transfected in H1650 cells, which indicated that both miR-126 vectors significantly increased expression of caspase 3 in H1650 cells (^*∗∗*^*P* < 0.01, ^*∗∗∗*^*P* < 0.001, *n* = 4, Figure 2(d)). It was also found that both miR-126 vectors significantly increased expression of caspase 9 in H1650 cells (^*∗∗∗*^*P* < 0.001, *n* = 4, Figure 2(e)). The MTT assay indicated that two miR-126 vectors significantly decreased the growth of H1650 cells (^*∗∗∗*^*P* < 0.001, *n* = 6, Figure 2(f)). Collectively, it was confirmed that KD of miR-126 induced apoptosis of A549 and H1650 cells.

The article "Ginsenoside Rg1 Suppresses Non-Small-Cell Lung Cancer via MicroRNA-126-PI3K-AKT-mTOR Pathway" was retracted in 2023. Reasons: signs of a paper mill; compromised peer review; unreliable results or conclusions.

### 3.3. GS-Rg1 Inhibited Expression of miR-126 and Lung Cancer Growth

Since GS-Rg1 has been reported to exert inhibitory effects on many kinds of cancers. The effects of GS-Rg1 on miR-126 expression and growth of lung cancer cells were investigated. The dose of GS-Rg1 used in the presentation was based on previous studies [9, 10]. It was found that GS-Rg1 significantly inhibited the expression level of miR-126 in the A540 cell line (Figure 3(a), ^*∗*^*P* < 0.05, ^*∗∗*^*P* < 0.01). GS-Rg1 also promoted the expression level of apoptosis markers including caspase 3 (Figure 3(b), ^*∗*^*P* < 0.05, ^*∗∗*^*P* < 0.01) and caspase 9 (Figure 3(c), ^*∗*^*P* < 0.05) in the A540 cell line. It was also found that GS-Rg1 significantly inhibited cell viability of A549 cells (Figure 3(d), ^*∗*^*P* < 0.05, ^*∗∗*^*P* < 0.01, ^*∗∗∗*^*P* < 0.001). Moreover, it was found that GS-Rg1 significantly inhibited the expression level of miR-126 in the H1650 cell line (Figure 3(e), ^*∗*^*P* < 0.05). GS-Rg1 promoted the expression level of apoptosis markers including caspase 3 (Figure 3(f), ^*∗*^*P* < 0.05) and caspase 9 (Figure 3(g), ^*∗*^*P* < 0.05) in the H1650 cell line. It was also found that GS-Rg1 significantly inhibited cell viability of H1650 cells (Figure 3(d), ^*∗*^*P* < 0.05, ^*∗∗*^*P* < 0.01, ^*∗∗∗*^*P* < 0.001). Taken together, it was demonstrated that GS-Rg1 could inhibit the expression level of miR-126 and the growth of lung cancer cells.

The article "Ginsenoside Rg1 Suppresses Non-Small-Cell Lung Cancer via MicroRNA-126-PI3K-AKT-mTOR Pathway" was retracted in 2023. Reasons: signs of a paper mill; compromised peer review; unreliable results or conclusions.

### 3.4. miR-126 Targets PIK3R2 and PI3K/mTOR Signaling in Lung Cancer Cells

The functions of miRNAs are elucidated with analyses of the genes they target. PIK3R2 was identified as a putative target of miR-126 using target prediction programs (TargetScan 7.2, https://www.targetscan.org/vert_72/) (Figure 3(a)). To further investigate the interaction of miR-126 and PI3K/mTOR signaling, the effects of miR-126 on elements of mTOR signaling were studied using WB. It was found that KD of miR-126 could increase protein level of phospharylated PI3K and mTOR in both A549 (Figure 3(b)) and H1650 cells (Figure 3(c)), while KD of miR-126 did not change protein level of total PI3K and mTOR in both A549 (Figure 3(b)) and H1650 cells (Figure 3(c)). Interestingly, it was found that phospharylated PIK3 was higher in non-small-cell lung cancer tissue (Figure 4(a)) than in paracancerous tissue (Figure 4(b)). Thus, we confirmed that miR-126 could interact with mTOR signaling in lung cancer cells.

### 3.5. Blocking PI3K Compromised Increase of miR-126 KD on Apoptosis in Lung Cancer Cells

To investigate the mechanism of action (MOA) of effects of miR-126 KD on apoptosis in lung cancer cells, two si-PI3KR2 vectors and si-scramble vectors were transfected in A549 cells, which indicated that two si-PI3KR2 vectors significantly decreased mRNA expression of PI3KR2 in A549 cells (^*∗∗*^*P* < 0.01, ^*∗∗∗*^*P* < 0.001, *n* = 4, Figure 5(a)). Interestingly, it was found that KD of PI3KR2 compromised increase of miR-126 KD on increase of caspase 3 mRNA expression in A549 cells (^*∗∗*^*P* < 0.01, *n* = 4, Figure 5(b)). In parallel, it was found that KD of PI3KR2 compromised increase of miR-126 KD on increase of caspase 9 mRNA expression in A549 cells (^*∗∗*^*P* < 0.01, ^*∗∗∗*^*P* < 0.001, *n* = 4, Figure 5(c)). Moreover, it was found that KD of PI3KR2 compromised increase of miR-126 KD on decrease of cell viability in A549 cells (^*∗∗*^*P* < 0.01, ^*∗∗∗*^*P* < 0.001, *n* = 4, Figure 5(d)). To further investigate, two si-PI3KR2 vectors and si-scramble vectors were transfected in H1650 cells, which indicated that two si-PI3KR2 vectors significantly decreased mRNA expression of PI3KR2 in H1650 cells (^*∗∗*^*P* < 0.01, ^*∗∗∗*^*P* < 0.001, *n* = 4, Figure 5(e)). Interestingly, it was found that KD of PI3KR2 compromised increase of miR-126 KD on increase of caspase 3 mRNA expression in H1650 cells (^*∗∗*^*P* < 0.01, ^*∗∗∗*^*P* < 0.001, *n* = 4, Figure 5(f)). In parallel, it was found that KD of PI3KR2 compromised increase of miR-126 KD on increase of caspase 9 mRNA expression in H1650 cells (^*∗∗*^*P* < 0.01, *n* = 4, Figure 5(g)). KD of PI3KR2 compromised increase of miR-126 KD on decrease of cell viability in H1650 cells (^*∗∗*^*P* < 0.01, ^*∗∗∗*^*P* < 0.001, *n* = 4, Figure 5(h)). Collectively, it was demonstrated that blocking PI3K compromised increase of miR-126 KD on apoptosis in lung cancer cells.

The article "Ginsenoside Rg1 Suppresses Non-Small-Cell Lung Cancer via MicroRNA-126-PI3K-AKT-mTOR Pathway" was retracted in 2023. Reasons: signs of a paper mill; compromised peer review; unreliable results or conclusions.

### 3.6. Blocking mTOR Compromised Increase of miR-126 KD on Apoptosis in Lung Cancer Cells

To further explore the effects of mTOR signaling on the increase of miR-126 KD on apoptosis in lung cancer cells, two si-mTOR vectors and si-scramble vectors were transfected in A549 cells, which indicated that two si-mTOR vectors significantly decreased mRNA expression of PI3KR2 in A549 cells (^*∗∗*^*P* < 0.01, ^*∗∗∗*^*P* < 0.001, *n* = 4, Figure 6(a)). It was found that KD of mTOR compromised increase of miR-126 KD on increase of caspase 3 mRNA expression in A549 cells (^*∗*^*P* < 0.05, ^*∗∗*^*P* < 0.01, *n* = 4, Figure 6(b)). Moreover, it was found that KD of mTOR compromised increase of miR-126 KD on increase of caspase 9 mRNA expression in A549 cells (^*∗*^*P* < 0.05, ^*∗∗*^*P* < 0.01, ^*∗∗∗*^*P* < 0.001, *n* = 4, Figure 6(c)). It was also found that KD of mTOR compromised increase of miR-126 KD on decrease of cell viability in A549 cells (^*∗*^*P* < 0.5, ^*∗∗*^*P* < 0.01, *n* = 4, Figure 6(d)). To further investigate, two si-mTOR vectors and si-scramble vectors were transfected in H1650 cells, which indicated that two si-mTOR vectors significantly decreased mRNA expression of mTOR in H1650 cells (^*∗∗*^*P* < 0.01, *n* = 4, Figure 6(e)). Interestingly, it was found that KD of mTOR compromised increase of miR-126 KD on increase of caspase 3 mRNA expression in H1650 cells (^*∗*^*P* < 0.05, ^*∗∗*^*P* < 0.01, *n* = 4, Figure 6(f)). In parallel, it was found that KD of mTOR compromised increase of miR-126 KD on increase of caspase 9 mRNA expression in H1650 cells (^*∗*^*P* < 0.05, *n* = 4, Figure 6(g)). KD of mTOR compromised increase of miR-126 KD on decrease of cell viability in H1650 cells (^*∗∗*^*P* < 0.01, ^*∗∗∗*^*P* < 0.001, *n* = 4, Figure 6(h)). Collectively, it was demonstrated that mTOR is closely involved in increase of miR-126 KD on apoptosis in lung cancer cells.

### 3.7. GS-Rg1 Inhibited Lung Cancer Growth via miR-126 and mTOR

In order to investigate the underlying mechanisms of the effects of GS-Rg1 on the growth of lung cancer cells, the A549 cell line was cotreated with GS-Rg1 and miR-126 inhibitor, which indicated that miR-126 inhibitor stopped the increased expression level of caspase 3 induced by GS-Rg1 in the A549 cell line (Figure 7(a), ^*∗*^*P* < 0.05) and H1650 cell line (Figure 7(b), ^*∗*^*P* < 0.05, ^*∗∗*^*P* < 0.01). Interesting, it was found that si-mTOR stopped increased the expression level of caspase 3 induced by GS-Rg1 in the A549 cell line (Figure 7(c), ^*∗∗*^*P* < 0.01) and the H1650 cell line (Figure 7(d), ^*∗*^*P* < 0.05, ^*∗∗*^*P* < 0.01). Thus, it was demonstrated that GS-Rg1 could inhibit lung cancer growth via miR-126 and mTOR.

The article "Ginsenoside Rg1 Suppresses Non-Small-Cell Lung Cancer via MicroRNA-126-PI3K-AKT-mTOR Pathway" was retracted in 2023. Reasons: signs of a paper mill; compromised peer review; unreliable results or conclusions.

## 4. Discussion

Increasing evidence indicates that the number of NSCLC patients is increasing in the world. A better understanding regarding NSCLC potentiates the discovery of effective therapies treating the disease. To investigate the role of miR-126 on the pathogenesis of NSCLC, it was the first to investigate miR-126 expression in NSCLC patients. Two NSCLC cells including A549 and H1650 cell lines were used. It was found that expression of miR126 was decreased in the PBMC of NSCLC patients compared to healthy controls. Expression of miR126 was decreased in cancer tissue compared to paracancerous tissues in NSCLC patients. GS-Rg1 significantly inhibited expression of miR126 and the growth of lung cancers. miR-126 KD remarkably increased expression of apoptosis genes including caspase 3 and caspase 9 and decreased cell viability in lung cancer cells including A549 and H1650 cells. Interestingly, *in Silico* analysis indicated that miR-126 could target the PI3K signaling pathway, which was confirmed by the WB assay. KD of PI3KR2 compromised promotion of miR-126 on cell apoptosis. Similarly, it was found that KD of mTOR compromised promotion of miR-126 on cell apoptosis. Finally, it was demonstrated that inhibition of GS-Rg1 on the growth of lung cancer cells was through miR-126 and mTOR. Thus, the present study indicated that GS-Rg1 may be a potential therapy for treating lung cancer.

According to the global cancer observatory (GCO), lung cancer is the deadliest form of cancer in the world, which causes a large population of deaths [21]. Understanding the pathogenesis of the disease plays an important role in the discovery of effective drugs to treat NSCLC. Seeking an effective biomarker is important to reduce the incidence rate of NSCLC. Several genes, including bromodomain PHD finger transcription factor (BPTF) [22], serum thrombospondin-2 [23], CTAPIII/CXCL7 [24], c-MET [25], and so on, have been reported to be biomarkers of NSCLC. Accumulating evidence indicates that miRNAs can be biomarkers of NSCLC. For example, Sui et al. found that miRNA-30 plays an important role in NSCLC and might be a biomarker for NSCLC [26]. Luo et al. confirmed that increased plasma miRNA-30a could be a biomarker for NSCCLC [27]. Circulating microRNA-590-5p was found to serve as a liquid biopsy marker in NSCLC [28]. Interestingly, the present study found that expression of miR-126 was decreased in the PBMC of NSCLC patients compared to healthy control. Expression of miR-126 was decreased in cancer tissue compared to paracancerous tissues in NSCLC patients (Figure 1). Moreover, it was found that miR-126 KD remarkably increased expression of apoptosis genes including caspase 3 and caspase 9 and decreased cell viability in lung cancer cells including A549 and H1650 cells in our study (Figure 2). In parallel, Santarelli et al. found that exosomal miR-126 was a circulating biomarker and was closely involved in regulating cancer progression in NSCLC [29]. Zheng et al. found that bone marrow mesenchymal stem cell-derived exosomal microRNA-126-3p inhibited the growth and process of pancreatic cancer by targeting ADAM9 [30]. Zhu et al. found that downregulated serum miR-126 was closely linked to aggressive progression and poor prognosis of gastric cancer [31]. Collectively, miR126 plays an essential role in the diagnosis of NSCLC.

The article "Ginsenoside Rg1 Suppresses Non-Small-Cell Lung Cancer via MicroRNA-126-PI3K-AKT-mTOR Pathway" was retracted in 2023. Reasons: signs of a paper mill; compromised peer review; unreliable results or conclusions.

GS-Rg1 has been broadly confirmed to exert an essential role in treating cancer [10]. For instance, Yu et al. found that GS-Rg1 could induce apoptosis in a caspase-independent manner in human lung cancer cells [32]. Consistently, in the present study, it was found that GS-Rg1 significantly decreased the growth of lung cancer cells (Figure 3). Interestingly, we also found that GS-Rg1 significantly decreased expression of miR-126 (Figure 3). Previous studies also demonstrated that GS-Rg1 had an influence on miRNAs [33, 34].

miR-126 was confirmed to involve in multiple signaling pathways such as angiogenic signaling, AKT/Rac1 signaling pathway, PI3K/AKT signaling pathway, SIRT1/Nrf2 signaling pathway, and so on [35]. The PI3K/ATK/mTOR pathway was confirmed to involve in pathogenesis of NSCLC [36]. In the present study, bioinformatics found that PI3KR2 was the target gene of miR-126 (Figure 4). Moreover, it was found that miR126 vectors increased phosphorylation of PI3K and mTOR in A549 and H1650 cells (Figure 4). Similarly, Cheng et al. found that LncRNA-XIST/microRNA-126 could be involved in cell proliferation and glucose metabolism via the IRS1/PI3K/Akt pathway in glioma [37]. Lin et al. found that miR-126 played an important role in the pathogenesis of glioma via regulating PTEN/PI3K/Akt and MDM2-p53 pathways [38]. Yang et al. found the maturation of miR-126-5p promotes ovarian cancer progression and could aid ovarian cancer progression through the PTEN-mediated PI3K/Akt/mTOR pathway [39]. Of note, it was found that KD of PI3KR2 compromised promotion effects of miR-126 on apoptosis of A549 and H1650 cells (Figure 6). Similarly, we also found that KD of mTOR compromised promotion effects of miR-126 KD on apoptosis of A549 and H1650 cells (Figure 8). Finally, we confirmed that the effects of GS-Rg1 on the growth of lung cancer cells were through miR-126 and mTOR (Figure 7). Thus, it is clearly confirmed that GS-Rg1 could inhibit the growth of lung cancer cells via the miR-126/PI3K/mTOR signaling pathway.

The article "Ginsenoside Rg1 Suppresses Non-Small-Cell Lung Cancer via MicroRNA-126-PI3K-AKT-mTOR Pathway" was retracted in 2023. Reasons: signs of a paper mill; compromised peer review; unreliable results or conclusions.

In conclusion, the present study confirms that GS-Rg1 could significantly inhibit the growth of lung cancer cells and the expression level of miR-126. Moreover, expression of miR-126 is reduced in lung cancer patients. KD of miR-126 could induce apoptosis of lung cancer cells. Importantly, it is found that miR-126 could target PI3KR2, and miR-126 could increase the protein level of phosphorylated PI3K and mTOR. The KD of PI3KR2 and mTOR weakens the promotion of miR-126 KD on apoptosis of A549 and H1650 cells. The effects of GS-Rg1 on the growth of lung cancer cells were through miR-126 and mTOR. In summary, the study confirms that GS-Rg1 significantly suppresses the growth of lung cancer cells, which might be developed into a therapeutic tool against lung cancer.

## Figures and Tables

**Figure 1:** The expression of miR-126 was downregulated in PBMC and lung tissue of NSCLC patients. (a) The expression of miR-126 was significantly lower in NSCLC compared to health control (*P* < 0.001, *n* = 81); (b) expression of the miR-126 was significantly higher in lung cancer tissues than lung paracancerous tissues (*P* < 0.001, *n* = 30).

**Figure 2:** Knockdown (KD) of miR-126 induced apoptosis of A549 and H1650 cells. (a) Two miR-126 vectors (#1 and #2) significantly increased expression of the caspase 3 in A549 cells (^*∗∗*^*P* < 0.01, *n* = 4); (b) both miR-126 vectors significantly increased expression of the caspase 9 in A549 cells (^*∗∗*^*P* < 0.01, *n* = 4); (c) two miR-126 vectors significantly decreased growth of A549 cells (^*∗∗∗*^*P* < 0.001); (d) both miR-126 vectors significantly increased expression of the caspase 3 in H1650 cells (^*∗∗*^*P* < 0.01, ^*∗∗∗*^*P* < 0.001, *n* = 4); (e) both miR-126 vectors significantly increased expression of the caspase 9 in H1650 cells (^*∗∗∗*^*P* < 0.001, *n* = 4); (f) two miR-126 vectors significantly decreased growth of H1650 cells (^*∗∗∗*^*P* < 0.001, *n* = 6).

**Figure 3:** GS-Rg1 inhibited expression of miR-126 and lung cancer growth. (a) GS-Rg1 significantly inhibited the expression level of miR-126 in A540 cell line (^*∗*^*P* < 0.05, ^*∗∗*^*P* < 0.01); (b) GS-Rg1 promoted the expression level of caspase 3 in the A540 cell line (^*∗*^*P* < 0.05); (c) GS-Rg1 promoted the expression level of caspase 9 in the A540 cell line (^*∗*^*P* < 0.05); (d) GS-Rg1 significantly inhibited cell viability of A549 cells (^*∗*^*P* < 0.05, ^*∗∗*^*P* < 0.01, ^*∗∗∗*^*P* < 0.001); (e) GS-Rg1 significantly inhibited the expression level of miR-126 in the H1650 cell line (^*∗*^*P* < 0.05); (f) GS-Rg1 promoted the expression level of caspase 3 in H1650 cell line (^*∗*^*P* < 0.05); (g) GS-Rg1 promoted the expression level of caspase 9 in the H1650 cell line (^*∗*^*P* < 0.05); (h) GS-Rg1 significantly inhibited cell viability of A549 cells (^*∗∗*^*P* < 0.01, ^*∗∗∗*^*P* < 0.001).

The article "Ginsenoside Rg1 Suppresses Non-Small-Cell Lung Cancer via MicroRNA-126-PI3K-AKT-mTOR Pathway" was retracted in 2023. Reasons: signs of a paper mill; compromised peer review; unreliable results or conclusions.

**Figure 4:** miR-126 targets PIK3R2 and PI3K/mTOR signaling in lung cancer cells. (a) The functions of miRNAs are elucidated with analyses of the genes they target. PIK3R2 was identified as a putative target of miR-126; (b) KD of miR-126 could increase the protein level of phospharylated PI3K and mTOR, but not the protein level of total PI3K and mTOR in A549 cells; (c) KD of miR-126 could increase the protein level of phospharylated PI3K and mTOR, but not the protein level of total PI3K and mTOR in H1650 cells.

**Figure 5:** Phospho-PI3K level was increased in non-small-cell lung cancer tissue than paracancerous tissue. (a) Phospho-PI3K staining in paracancerous tissue; (b) phospho-PI3K staining in non-small-cell lung cancer tissue.

**Figure 6:** Blocking PI3K compromised increase of miR-126 KD on apoptosis in lung cancer cells. (a) Two si-PI3KR2 vectors significantly decreased mRNA expression of PI3KR2 in A549 cells (^*∗∗*^*P* < 0.01, ^*∗∗∗*^*P* < 0.001, *n* = 4); (b) KD of PI3KR2 compromised increase of miR-126 KD on increase of caspase 3 mRNA expression in A549 cells (^*∗∗*^*P* < 0.01, *n* = 4); (c) KD of PI3KR2 compromised increase of miR-126 KD on increase of caspase 9 mRNA expression in A549 cells (^*∗∗*^*P* < 0.01, ^*∗∗∗*^*P* < 0.001, *n* = 4); (d) KD of PI3KR2 compromised increase of miR-126 KD on decrease of cell viability in A549 cells (^*∗∗*^*P* < 0.01, ^*∗∗∗*^*P* < 0.001, *n* = 4); (e) two si-PI3KR2 vectors and si-scramble vectors were transfected in H1650 cells, which indicated that two si-PI3KR2 vectors significantly decreased mRNA expression of PI3KR2 in H1650 cells (^*∗∗*^*P* < 0.01, ^*∗∗∗*^*P* < 0.001, *n* = 4); (f) KD of PI3KR2 compromised increase of miR-126 KD on increase of caspase 3 mRNA expression in H1650 cells (^*∗∗*^*P* < 0.01, ^*∗∗∗*^*P* < 0.001, *n* = 4); (g) KD of PI3KR2 compromised increase of miR-126 KD on increase of caspase 9 mRNA expression in H1650 cells (^*∗∗*^*P* < 0.01, *n* = 4); (h) KD of PI3KR2 compromised increase of miR-126 KD on decrease of cell viability in H1650 cells (^*∗∗*^*P* < 0.01, ^*∗∗∗*^*P* < 0.001, *n* = 4).

**Figure 7:** Blocking mTOR compromised increase of miR-126 KD on apoptosis in lung cancer cells. (a) Two si-mTOR vectors significantly decreased mRNA expression of PI3KR2 in A549 cells (^*∗∗*^*P* < 0.01, ^*∗∗∗*^*P* < 0.001, *n* = 4); (b) KD of mTOR compromised increase of miR-126 KD on increase of caspase 3 mRNA expression in A549 cells (^*∗*^*P* < 0.05, ^*∗∗*^*P* < 0.01, *n* = 4); (c) KD of mTOR compromised increase of miR-126 KD on increase of caspase 9 mRNA expression in A549 cells (^*∗*^*P* < 0.05, ^*∗∗*^*P* < 0.01, ^*∗∗∗*^*P* < 0.001, *n* = 4); (d) KD of mTOR compromised increase of miR-126 KD on decrease of cell viability in A549 cells (^*∗*^*P* < 0.5, ^*∗∗*^*P* < 0.01, *n* = 4); (e) two si-mTOR vectors significantly decreased mRNA expression of mTOR in H1650 cells (^*∗∗*^*P* < 0.01, *n* = 4); (f) KD of mTOR compromised increase of miR-126 KD on increase of caspase 3 mRNA expression in H1650 cells (^*∗*^*P* < 0.05, ^*∗∗*^*P* < 0.01, *n* = 4); (g) KD of mTOR compromised increase of miR-126 KD on increase of caspase 9 mRNA expression in H1650 cells (^*∗*^*P* < 0.05, *n* = 4); (h) KD of mTOR compromised increase of miR-126 KD on decrease of cell viability in H1650 cells (^*∗∗*^*P* < 0.01, ^*∗∗∗*^*P* < 0.001, *n* = 4).

The article "Ginsenoside Rg1 Suppresses Non-Small-Cell Lung Cancer via MicroRNA-126-PI3K-AKT-mTOR Pathway" was retracted in 2023. Reasons: signs of a paper mill; compromised peer review; unreliable results or conclusions.

**Figure 8:** GS-Rg1 inhibited lung cancer growth via miR126 and mTOR. (a) miR126 inhibitor stopped increased the expression level of caspase 3 induced by GS-Rg1 in A549 cell line (^*∗*^*P* < 0.05); (b) miR126 inhibitor stopped increased the expression level of caspase 3 induced by GS-Rg1 in H1650 cell line (^*∗*^*P* < 0.05, ^*∗∗*^*P* < 0.01); (c) si-mTOR stopped increased the expression level of caspase 3 induced by GS-Rg1 in A549 cell line (^*∗∗*^*P* < 0.01); (d) si-mTOR stopped increased the expression level of caspase 3 induced by GS-Rg1 in H1650 cell line (^*∗*^*P* < 0.05, ^*∗∗*^*P* < 0.01).

**Table 1:** Primers used in the study.

Genes		Sequence		GC%
PI3KR2	Sense	GAGACCAGTACCTCGTGTGG	119	60
	Antisense	ATCGTCCTCGTCCTCCATGA		55
mTOR	Sense	CTTAGAGGACAGCGGGGAAG	111	60
	Antisense	TCCTTTAATATTCGCGCGGC		50
miR-126	Sense	CGCTGGTGATGGGACATTATT	84	48
	Antisense	GCTGTGGACAGCGCATTATT		50

## Data Availability

The authors confirm that the data supporting the findings of this study are available within the article.
